The article "Human-in-the-Loop Predictive Analytics Using Statistical Learning" was published in 2021. Journal: J Healthc Eng.

# Human-in-the-Loop Predictive Analytics Using Statistical Learning

**DOI:** 10.1155/2021/9955635

**Published:** 2021-07-29

**Authors:** Anusha Ganesan, Anand Paul, Ganesan Nagabushnam, Malik Junaid Jami Gul

**Affiliations:** The School of Computer Science and Engineering, Kyungpook National University, Daegu, Republic of Korea

## Abstract

The human-in-the-loop cyber-physical system provides numerous solutions for the challenges faced by the doctors or medical practitioners. There is a linear trend of advancement and automation in the medical field for the early diagnosis of several diseases. One of the critical and challenging diseases in the medical field is coma. In the medical research field, currently, the prediction of these diseases is performed only using the data gathered from the devices only; however, the human's input is much essential to accurately understand their health condition to take appropriate decision on time. Therefore, we have proposed a healthcare framework involving the concept of artificial intelligence in the human-in- the-loop cyber-physical system. This model works via a response loop in which the human's intention is concluded by gathering biological signals and context data, and then, the decision is interpreted to a system action that is recognizable to the human in the physical environment, thereby completing the loop. In this paper, we have designed a model for early prognosis of coma using the electroencephalogram dataset. In the proposed approach, we have achieved the best results using a statistical learning algorithm called autoregressive integrated moving average in comparison to artificial neural networks and long short-term memory models. In order to measure the efficiency of our model, we have used the root mean squared error (RMSE), mean absolute error (MAE), and mean squared error (MSE) value to evaluate the linear models as it gives the difference between the measured value and true or correct value. We have achieved the least possible error value for our dataset. To conduct this experiment, we used the dataset available in the phsyionet opensource community.

## 1. Introduction

Humans are miraculous as our intellectual capabilities and strengths support us greatly to discover, create, and improvise a diversity of tools, processes, and technologically advanced devices to create a smooth and comfortable life on the Earth for everyone. In recent years also, we have accomplished many creative discoveries and advancements using the developing technology in the area of computer science, healthcare, transportation, and networking, and most of them are remarkable due to their benefits for human life and the way they have drastically changed our lives. Likewise, there are several major challenges in the field of biomedical that involves the interpretation of human intentions under the physical environment. These problems could be solved or improvised by the Human-in-the-Loop Cyber-Physical System (HiLCPS) concept.

The idea of the HiLCPS emphasizes on executing more intellectual thoughts using Brain-Computer Interaction (BCI) characteristics [1, 2]. HiLCPS supports decision making promptly with historical observations on the interaction amongst the human and physical environment or circumstance. This is also advantageous in the medical field to overcome the challenges encountered during the diagnosis of any disease. In order to understand the concept of HiLCPS, the origin of the Cyber-Physical System (CPS) has to be studied. Even recent research studies have highlighted the significance of CPS in Artificial Intelligence (AI) [3]. The CPS can sense and control the environment with a network of devices that works towards shared goals. It supports the unification of robotics and wireless sensors networks [4, 5]. Thus, when integrating the cyber-physical system for human-computer interaction, it creates value to artificial intelligence learning from the human cognition perspective rather than relying on the feedback from the connected devices only. The recent efforts to monitor the rapid-spreading pandemic COVID-19 also prove that relying only on computer data was ineffective. So, the input from human and connected devices is integrated with the decision-making loop to make proactive actions towards human well-being. Therefore, in this paper, we have proposed an architecture for healthcare and made a prediction model for coma with the integration of HiLCPS and AI. As the human brain is the most vital organ, we decided to make a prediction model for one of the critical diseases affecting the human brain. Coma derives its meaning from a Greek word “deep sleep.” Coma is a sleep-like condition when the patients are totally unresponsive and are unable to get back to the normal condition. Biologically, coma is induced when the brain stem is affected. The brain stem manages the spontaneous and unconscious controls which are called vegetative functions of the body that include the heart rate, blood pressure, body temperature, and breathing [6]. Around 18% of comatose patients reach the death stage. Hence, it is a critical condition of the human brain.  Figure 1 shows some inducing factors and consequences faced due to the comatose condition.

There is a chance of continuous coma after anesthesia in certain patients. There can be several causes for the prolonged recovery from anesthesia for patients. The factors could be related to the patient's health condition, pharmacological and surgical reasons, or even due to drug overconsume [7]. Anesthesia specialists must be aware of mysteriously delayed recovery scenarios that can happen due to preexisting health issues [8, 9]. Due to drug overdose, the coma can mostly lead to a fatal state for a person [10, 11]. At the same time, there are benefits from coma as well; one such is that the pharmacologically induced coma supports for treatment to certain health problems such as Refractory Status Epilepticus (RSE) [12]. Coma can be predicted using the changes observed in the EEG and ECG patterns of a human being. They also serve as a good source of input to identify the onset of coma in a human. Our main aim in this paper is to design a proposed architecture for healthcare by making use of the benefits from the HiLCPS framework and AI as there is a vital necessity for involving human's interaction to the environment and cognitive intentions along with the data gathered from the sensor network to take a better proactive decision in the process of healthcare monitoring. While we rely only on the data gathered from devices, there can be chances of misinterpretation of the data. Human's input is more essential to understand the current health condition in a much accurate way.

In the proposed system, we used EEG data taken from an open-source database and performed the experimental analysis with ARIMA and compared the results with ANN and LSTM models to measure the effectiveness of our model. As a result of our experiment, the ARIMA model was observed to be the best technique to handle these statistical data that takes less computational power than other machine learning or deep learning algorithms. To evaluate our experiment results, we have considered the performance metrics such as mean absolute error (MAE), mean squared error (MSE), and root mean squared error (RMSE).

The rest of this paper is organized as follows.  Section 2 provides literature review about the cyber-physical system and human-machine interface with EEG signal prediction and gives better understanding of HiLCPS.  Section 3 gives insight about the patterns of the electroencephalogram and electrocardiogram in a normal person and coma person that have been used for identifying the difference in EEG signals to predict coma.  Section 4 provides the materials and methods that were used in conducting this study.  Section 5 details about the proposed architecture and gives explanation about integration of artificial intelligence and the human-in-the-loop concept.  Section 6 provides information about the experiments and discusses the results that are observed. Finally, we have concluded with the highlights of the study performed.

## 2. Literature Review

Cyber-Physical Systems (CPSs) are the systems that integrate the physical environment with the computational environment with the sensors and networking technologies available [13]. Sensors are key devices that facilitate collecting of data from real-time situations, manage the data collected in a digital structure, and spread it to the physical environment using the Internet [14]. It combines these sensors and the computational abilities of the devices to achieve the expected results. For example, it can support remote monitoring of personal health conditions. Healthcare systems achieved more benefits such as deals well with new and unpredictable surroundings, network integration, good interaction between human and systems, and fast response time using this concept [15–17]. The CPS using the brain-computer interface brought some alternate solutions for health issues of physically challenged and elderly persons as the BCI is an advanced technology that creates a human interaction with the externally available electronic and electromechanical equipment related to encoding and decoding of brain electrical signals. It is also helpful for humans having cerebral palsy, which is brain and muscle weakness or problems [18]. Many Russian researchers have conducted many experiments, and results revealed that the BCI based on EEG signals is much helpful in recognizing the human mental commands using the P300 waves. P300 (P3) waves are event-related potential constituents that induce the decision-making process, and they are regarded as an endogenous potential, since their presence connects not to the physical attributes of a stimulus but also to an individual's reaction to it. These waves are observed in a time-locked interval appearing as a positivity for 300 to 400 ms after the stimulus presentation. Time interval ranges from 250 ms to 900 ms in a wide-spread manner with an amplitude of minimum 5 *μ*V to 20 *μ*V for audio and visual stimulated potential [19]. There was an experiment performed with humans who had extreme neuromuscular disorder, yet they were able to obtain and retain control over evident patterns of EEG signals and utilize the same to control the external devices. Patients were asked to visualize or make a movement of their hands or feet by the form of the corresponding object. This experiment remarked as the first evidence for integration between the BCI from EEG and the physical environmental control system [20]. Hence, the CPS using the BCI helped the healthcare industry to make alternate solutions for certain health problems. There is some literature about the scope of EEG in the CPS [21]. EEG is a test to detect the electrical signals in the human brain using small metallic discs or electrodes placed in the human scalp. This is a noninvasive and much economical technology that has an effective ability for creating BCIs. EEG (electroencephalography) is the most generally used method for diagnosing neural diseases such as stroke, epilepsy, coma, and Alzheimer's disease.

In the literature, the proposed system for the detection of stroke is based on the wearable wireless QEEG devices which were used for EEG recording. The system interacts between the sensors in these devices and computational set up using the wireless network for stroke detection. Thus, EEG signals taken from the sensors are a component to support the function of the cyber-physical system for interacting between the physical world and the computational world. With the rapid development of sensing technologies, the benefits contributed by this concept, the innovative idea of introducing the human-in-the-loop cyber-physical system was evolved. However, Industry 4.0 highlighted the requirements to have such a tight interaction between the CPS and the humans: (1) good and clear bidirectional information flow and (2) a proper, interactive human-machine interface (HMI) [22]. Many kinds of literature have explained the enrichment of this concept. It is a model that supports data and decision-making intelligence. The theory of HiLCPS is to emphasize the human's intention, feelings, psychological situations, and actions in the sensors and finally incorporate the information collected to the control loop as a result to discover the working of the cyber-physical system [23]. The presence of humans in the control loop creates a massive change in reliability and performance. Therefore, HiLCPS is much consistent in monitoring human activities which is very interminable [24]. On the other hand, there are several literature works which highlight the health condition prediction using statistical and deep learning algorithms such as ARIMA, ANN, and LSTM. In [25], the authors have used for healthcare decision-making process; however, it is strange to notice that there were certain limitations of the model due to the structure complexity of ANN architecture and the authors must be aware of the complex nature of the network to get the fundamental understanding of the architecture. In [26], the authors have deployed an LSTM model for predicting healthcare trajectories from medical records. Here, the authors have introduced a DeepCare end-to-end deep dynamic memory neural network for personalized healthcare using LSTM. However, there are other advanced algorithms that can account for temporal models in irregular timing. Hence, we have proposed an architecture that integrates the human-in-the-loop cyber-physical system with Artificial Intelligence (AI) using these statistical and deep learning algorithms to make a better decision-making model for the wellness of a human being.

## 3. Electroencephalogram and Electrocardiogram Patterns in a Normal Person and Coma Person

The patterns of EEG and ECG help in predicting the onset of coma. The variations observed in the patterns of these signals help classifying between the normal EEG and ECG signals and the coma EEG and ECG signals.

### 3.1. Electroencephalogram in a Normal Person

EEG data from the human brain comprises of mainly 4 types of background activity, namely, alpha, theta, delta, or beta. The frequency of these background activities generally ranges from 0 to 35 Hz. Each activity relates to the human condition such as awake or 4 sleep stages [27]. The explanation of this classification is given below based on the frequency of the waves.  Figure 2 gives the frequency bands for each type of activity in the EEG signal.

Delta waves ranging from 0 to 4 Hz are recorded with much lesser brain activities in deep sleep NREM stage 3. Theta waves ranging from 4 to 7 Hz are noted during NREM sleep stage 1 when there is drowsiness, muscle tone throughout the body starts to relax, and brain wave activity begins to slow down from that of the awake state. Alpha waves ranging from 7 to 13 Hz originate from the occipital lobes during awake relaxation, yet having higher amplitude on the leading side. Beta waves ranging from 13 to 35 Hz are connected to the awake period of humans such as consciousness, actions being performed while the eyes are open. There are also other two waves such as gamma and mu waves. Gamma waves range from 30 to 100 Hz, and these are generated by the different combinations of neurons in a neural network. Mu waves range from 8 to 13 Hz and reflect the mirror image of the neural activity.

These are found overlapping the alpha waves in EEG. The EEG recordings are correlated to the state of a human being with these 4 main brain activities in different patterns being observed. The theta waves increase during stage 1 NREM sleep. In stage 2 NREM sleep, there are sleep spindles of bandwidth 12–14 Hz and background waves from 3 to 6 Hz. Delta waves are observed during NREM stage 3 called deep sleep. As mentioned above, alpha and beta waves constitute the wakefulness period and REM sleep period, and the EEG patterns during these periods are similar.

Figure 3 shows the EEG patterns during all sleep stages and anesthesia sedation. The EEG patterns are different based on the age of humans because in the case of children and newborns, there is a dominant presence of slow-wave brain activity rather than the adults where rapid brain activity is prevailing. This happens due to brain maturity before describing the EEG patterns with the background activity which represents coma. Even the ECG patterns represent the stages of the sleep and wakefulness period in humans.

### 3.2. Electrocardiogram in a Normal Person

Electrocardiogram (ECG) is a novel method for cardiac analysis; it provides valuable evidence about the vital parts of the body concerning other human organs. To study the ECG patterns, we must know the parameters in ECG which help to distinguish the action performed by a human such as sleep and awake state. An initial electrical signal on a regular ECG generated from the atria that is called the *P* wave. Depolarization of the ventricles contributes to the major portion of the ECG; it is referred to as the *QRS* complex.

- The *Q* wave is the first preliminary downward or “negative” deflection
- The *R* wave is then the next upward deflection
- The *S* wave is then the next deflection downwards, provided it crosses the isoelectric line to become briefly negative before returning to the isoelectric baseline [30]

The interval measured from the onset of the *P* wave to the first refraction of the *QRS* complex is called a *PR* interval. The normal range for the *PR* interval is 120 to 200 ms. Heart Rate Variability (HRV) is another parameter. It is the oscillation in time intervals among the adjacent heartbeats. These consecutive intervals are called as Interbeat Intervals (IBIs). Heart rate oscillations are nonlinear and complex [31]. HRV is generated in combination with the heart-brain interactions and active autonomous nervous system processes. There have been several experiments and analyses made to assess the HRV under sleep stages 1–3 in NREM and REM sleep. One such analysis made at the Department of Veterans Affairs Medical Center, Wright University, explained how HRV impacts the stages of the sleep and awake state of a human [32]. The correlation between the EEG power range and HRV is clearly illustrated in some studies. It is said that HRV's highly normalized frequency is connected to the EEG power ranges that define the sleep stages [33, 34]. Corresponding changes in cardiac activity monitored by HRV frequency bring the changes in the delta waves in EEG. This correlation of electrocardiac waves to sleep stages is measured by the HRV analysis. This analysis involves assessing the period between two successive heartbeats. This interval is referred to as the *R-R* interval or *N*-*N* interval. Here, *R* is the peak condition of the *QRS* complex and *N* is the normal *R* peak. In an ECG wave, the waves which are disturbed by noise and other intrusions have the minimum amplitude. So, the wave which has the maximum amplitude is called the *R* peak. Despite that these waves will be changing in shape and amplitude due to noise being added, the highest amplitude waves keep remaining in the ECG pattern [35].  Figure 4 depicts the HRV analysis with the *R*-*R* interval to understand the stages of sleep.

### 3.3. Classification of EEG and ECG in a Coma Person

Coma is a period in which the frequencies of the brain activities in the EEG data define the state of the human brain. When the alpha activity has a frequency range from 8 to 13 Hz in unarousable individuals, it is called the alpha coma [37]. It is more visible in the frontal areas of the brain. This takes place typically owing to an overdose of drugs and consuming intoxicating drugs. The consequence of this kind of coma is very unfortunate as the fatal rate surpasses 90%. Theta coma arises while there is a transmission of unreactive theta waves, and it is frequently seen in the anterior parts of the brain. This coma mostly results in hypoxic-ischemic brain injury. Hypoxic-ischemic EEG wave patterns are normally observed in new-born babies whenever there is not sufficient oxygen and blood supplied to the infant's brain. It is the utmost risky state of the brain. Theta coma waves ultimately affect the fluctuations in the delta waves, thus causing brain death. Brain death is nonreversible damage to all brain activities, and it is also a state with no electrical signals and shows only an isoelectric flat line. Whereas even in a deep coma state, there can be EEG waves observed to an extent. Likewise, delta and beta activities even cause coma. In delta coma, the EEG patterns normally display a polymorphic shape and blunt triphase waves. It can be categorized into two types regarding the amplitude of the attained waves that is expressed in microvolts (*μ*V). At any time, the delta waves of bandwidth 1–3 Hz are recorded with an amplitude of several 100 *μ*V, which is called as high-voltage delta Coma. It commonly takes place in the advanced stages of coma. This also results in unfortunate situations. On the other hand, while the delta waves and theta waves are integrated into the EEG pattern with less amplitude under 20 *μ*V, it is known as low-voltage delta coma. This can take place even in healthy human beings. It is related to massive brain damage. Lastly, beta coma is highly reversible as it has a good probability of diagnosis. This coma occurs in individuals who consume intoxicated sedative drugs. With lesser intoxication period, the human can be recovered from this coma with appropriate medical treatment.  Figure 5 shows the difference in EEG patterns to know the type of coma concerning changes in the respective activity.

Description of how ECG data help identifying coma is given in [38]. A 66-year-old woman was taken to the emergency care unit in a hospital on an early morning. She was admitted with hyperventilation [39] that defines a state in which an individual begins to breathe faster than normal. Her medical history discloses that she was having manic or bipolar depression [40], a syndrome that occurs because of oscillations between opposite boundaries in a person's mood through high-level energy. Due to the drugs consumed for the depression, her ECG data indicate ventricular escape strike of 40 beats/min and widened *QRS* complexes at 0.24 s with RBBB (Right Bundle Branch Block) and LAFB (Left Anterior Fascicular Block) structures; then, they have discovered during her treatment that she had myocardial infraction as a result of extreme anaemia with an Hb count of 2.8 mmol/l and also intense stress [41]. This declines the blood flow to parts of the heart, thereby creating impairment to the heart muscles. As a final point, this disruption in the *QRS* complex on the ECG data caused the patient to enter the comatose period. On the other hand, she did make a progress along with right-arm paralysis.  Figure 6 shows the ECG patterns on coma.

## 4. Materials and Methods

The materials and methods used to perform the simulation to get the desired output are described below.

### 4.1. Materials

The simulation was performed in an environment setup using Python and a Python-integrated environment with TensorFlow and Keras libraries for statistical models' libraries to implement the models to create the prediction models.

### 4.2. Methods

The methods used for designing the proposed architecture and computation model are given below.

#### 4.2.1. Cyber-Physical System

The cyber-physical system in healthcare provides several applications such as elderly care and assisted living care. Its application in healthcare can be classified into two categories: (1) assisted and (2) controlled. In the assisted application, the CPS includes the health monitoring of a person remotely without disturbing the person's normal life. In the controlled application, the CPS interacts in a controlled environment with the hospital, intensive care, bedside monitors, biosensors, and so on to ensure the patient's condition improves and their safety at a place. The proposed architecture considers initially the assisted application of the cyber-physical system in healthcare for remotely monitoring, and in case of any emergency, the alert message is sent to the patient and once the patient is under a controlled environment, the CPS application moves to the controlled category. The CPS interacts with sensors in wearable devices to collect the EEG or ECG data from the human through the wireless sensor networks and transmits the sensing data to the storage network. From there, it is sent for the computation and intelligent decision-making system. Usually, the CPS in healthcare shares the computed result to the user via cellular or Wi-Fi network. But, this architecture involves human intervention from the consumer as well as healthcare specialist to analyze the computed result along with medical knowledge and expertise. Thus, we bring the concept of human-in-the-loop cyber-physical system to create a better decision-making model.

#### 4.2.2. Human-in-the-Loop Cyber-Physical System

The Human-in-the-Loop Cyber-Physical System (HiLCPS) comprises 3 parts: human, the embedded system (which is a cyber component), and the physical environment. The cyber component with the wireless sensors is boosting the communication from human to the physical environment. Using this concept, the architecture starts with the human who interacts with the physical environment using the cyber part that consists of sensors, wireless networks for communication, and also with the computation system of the cyber-physical system. This enables the human to make better decisions concerning the health condition. When the networked systems are closed with humans in the loop, it improves the medical workflows and patient safety. Integration of this concept with artificial intelligence, we have performed the computation of the input data. The belowmentioned statistical learning method was used in our experiment for the computation model.

#### 4.2.3. Autoregressive Integrated Moving Average Model

ARIMA means autoregressive integrated moving average. This is a grouping of prototypes or models that one details a certain time series arising from their prior values, in other words, its lags and also the postponed prediction errors; henceforward, with methods, we can figure out the expected imminent values [42, 43]. Moreover, a nonseasonally generated time series which demonstrates arrangements and remains to be subjective white noise can make use of this model. This ARIMA network can be defined with three labels as *p*, *d*, and *q*.

An Autoregressive (AR) model is a typical one where *Y*_t_ counts on its lags alone; here, “*Y*_*t*_ is termed to function for the lags in *Y*_*t*_.”

(1) $$\begin{array}{c} Y_{t}=\alpha +\beta_{1}Y_{t-1}+\beta_{2}Y_{t-2}+\cdots +\beta_{p}Y_{t-p}+\varepsilon_{1}. \end{array}$$

In equation (1), *Y*_*t*−1_ denotes the lag1 of the series, *β*_1_ represents the number of lags 1 that is derived from the model, and *α* refers to the intercept that is also resulting from the model.

Similarly, the Moving Average (MA) model is a typical one where *Y*_*t*_ counts on the lagged prediction errors.

(2) $$\begin{array}{c} Y_{t}=\alpha +\varepsilon_{t}+\phi_{1}\varepsilon_{t-1}+\phi_{2}\varepsilon_{t-2}+\cdots +\phi_{q}\varepsilon_{t-q}. \end{array}$$

In equation (2), the errors terms are the errors of the AR models of their lags. The *E*_*t*_ and *E*_(*t*−1)_ errors could be calculated using the following equations:

(3) $$\begin{array}{c} Y_{t}=\beta_{1}Y_{t-1}+\beta_{2}Y_{t-2}+\cdots +\beta_{0}Y_{0}+\varepsilon_{t},\\ Y_{t-1}=\beta_{1}Y_{t-2}+\beta_{2}Y_{t-3}+\cdots +\beta_{0}Y_{0}+\varepsilon_{t-1}. \end{array}$$

Hence, the description in equation (3) defines AR and MA models discretely.

ARIMA is a model in which the time series was differenced at the minimum one time to make it fixed. Subsequently, we combine the Autoregressive (AR) and Moving Average (MA) specifications from equations (1) and (2). Then, we have an equation as follows:

(4) $$\begin{array}{c} Y_{t}=\alpha +\beta_{1}Y_{t-1}+\beta_{2}Y_{t-2}+\cdots +\beta_{p}Y_{t-p}\varepsilon_{t}+\phi_{1}\varepsilon_{t-1}+\phi_{2}\varepsilon_{t-2}+\cdots +\phi_{q}\varepsilon_{t-q}. \end{array}$$

ARIMA workflow consists of model identification, parameter assessment, and diagnostic testing processes [24]. All these processes are reiterated to get the most suitable fitting model for prediction. This model empowers healthcare specialists to analyze and interpret a large health dataset to predict the factors that would impact the healthy life of a human. It also promotes preventive healthcare services, and giving the operationalization of this method can be effective for emergency readiness, health planning, and appropriate healthcare service. In the simulation experiment to evaluate the efficiency of the ARIMA model, we computed the results using ANN and LSTM for comparative analysis.  Figure 7 explains how the human, cyber system, and healthcare environment are integrated towards a closed loop for active monitoring of the human's health condition.

## 5. Proposed Architecture

Figure 8 shows the architecture which is designed to make a predictive model for identifying the onset of coma with the EEG and ECG data using AI.

There are 3 major layers in this architecture:

  (1) Consumer data generation and notification layer
  (2) Data processing and intelligence layer
  (3) Healthcare environment layer

### 5.1. Consumer Data Generation and Notification Layer

This layer deals with consumer data generation (input) and alert notification (output) of the architecture. In this layer, the data generation function is carried out, in which ECG and EEG data are collected via wearable devices and sensors for those who are enrolled in the healthcare system. Also, the alert notification from the healthcare environment happens in this layer in case of any necessity concerning the human's health.

### 5.2. Data Processing and Intelligence Layer

This layer is further classified into two sublayers:

  (1) Communication and data management layer
  (2) Computational intelligence layer

#### 5.2.1. Communication and Data Management Layer

In this layer, the data gathered are transmitted from the sensors in the wearable device by Wi-Fi or mobile data along with the Bluetooth technology to the data storage server in the cloud network. The successfully transmitted data such as EEG data from the brain can contain information about the teeth, eye movements, and so on. So, the data must undergo the data wrangling process, where the data transformation and data cleaning processes are performed to make the data clear and relevant for the predictive analysis. In the data transformation process, the data format is changed as suitable for this prediction model and also data quality check is performed after the formatting changes are being made to ensure that there is no effect on the data values due to the formatting modification. In the data cleaning process, the removal of outliers, null values, and corrupted values is carried out. Then, the structure of the data is fixed concerning the requirement for the model. As a result of the entire data wrangling process, we have clear preprocessed data that are stored in the cloud storage using any mode of network communication. Also, this layer is responsible for maintaining the historical data and creating a knowledge database that can support the computation of the data model.

#### 5.2.2. Computational Intelligence Layer

The preprocessed data are used for data modelling in this layer. This is the layer where the artificial intelligence plays a role in the training and testing of the model using the preprocessed data. This layer comprises the AI inference engine, which is accountable for the model deployment and performance monitoring activities and also helps to determine how effectively the AI technologies improvise the prediction accuracy and efficiency and solve real health problems. Thus, AI-aided diagnosis is much helpful for early prediction on any health issues. AI aiding has two main features: (1) it can handle an enormous amount of data promptly when compared to humans and (2) AI can improve accuracy through learning and analyzing huge data with a focus to find a solution or get a knowledge base or inference from the data. Hence, the preprocessed EEG data and ECG data are modelled using any of the AI to make the prediction model and perform some analyzing and learning from these data and apply logical reasoning and optimizing in identifying any abnormalities of the patterns observed in the EEG and ECG data that indicate the onset of coma for the human. Also, in case of any abnormalities on the data pattern observed, the healthcare specialist is notified with the data visualized using the network communication, and then, a medical analysis of the observations is made in the healthcare environment layer by the healthcare specialist or the doctor. Else, the output data are stored in the cloud network for historical maintenance of records and future learning by the AI model.

### 5.3. Healthcare Environment Layer

In this layer, the visualization of the predicted data is used as input to perform the medical analysis about the human's health condition. If there is an emergency requirement based on insight, an alert message will be received by the smart device through the communication and data management layer, which is a sublayer of the data processing and intelligence layer. Therefore, the healthcare environment layer includes the human and healthcare specialist as the end-users.

The architecture takes the input as EEG and ECG data taken from the human using the wearable device sensors which acts as a cyber-physical system, with a human's input (healthcare specialist and the human who has enrolled in the healthcare system). As the input is taken from the human and the computed output is fed back to the human, the loop is completed.

In our experiment, we have performed the simulation using ARIMA and compared with ANN and LSTM models, and we evaluated the models using the error prediction metrics. The simulation results were achieved using the statistical learning method, ARIMA, which was an easy and effective computation method and was useful in understanding the past or future data in a series. Also, it took less computation power. We achieved a best-fitting model using this method. EEG data which were a good source of information and the variations on the EEG data signals for coma helped in getting a good prediction model using ARIMA.

## 6. Results and Discussion

From the dataset taken from the open source [44], we performed our experiment with a setup using the hardware and software specifications as given in Table 1. Figures 9 and 10 represent the EEG data signal for normal sleep and coma, respectively. Based on the simulation, the results as shown in Figures 11 and 12 were achieved. For our simulation, we considered the ARIMA model for forecasting. The ARIMA model is a set comprising of models that defines a particular time set derived from its former values, especially its very own lags and deferred estimate errors; henceforth, it uses formulations to work out the expected upcoming values. AR (autoregressive) uses the relationship among the lagged observation and actual observation; “I” is meant for integrated which uses the differencing method to make the time series static, and MA (moving average) uses the dependency among the residual error and the observation. The sequence and residual plots of ARIMA help identifying the model structure such as AR model, MA model, or mixed.

To identify the best lags, we fitted several models with different lag choices, for instance, fit all combinations of *p*=1,…, 4 and *q* = 1,…, 4 (a total of 16 models) and store the loglikelihood objective function and number of coefficients for each fitted model.

Then, we calculate the BIC for each fitted model. The number of parameters in a model is *p* + *q* + 1 (for the AR and MA coefficients and constant term).

One way to do it is to use <auto. arima> to verify what the *p*, *d*, and *q* values. In other words, the lags and the values are automatically best fitted.

Another approach to obtain is to try a different model, for example, give an ARIMA model with the related *p* value.

1. ARIMA (0,0,1)
2. ARIMA (0,1,1)
3. ARIMA (1,0,0)
4. ARIMA (0,1,2)
5. ARIMA (1,0,1)
6. ARIMA (2,0,2)

The related RMSE values between models are calculated, and the best one was chosen. In our case, we had ARIMA (3,1,1), where AR = 3 is for autoregressive, *I* = 1 for integrated, and MA = 1 for moving average.

Figure 12 gives the prediction results, the blue line denoting the actual observations and the red line denoting the predicted values. The forecasted values in the red line match pretty close to the underlining true values in the blue line, and they are well within the confidence intervals of our forecast.  Figure 11 shows the ARIMA model result with the 153 observations using the css-mle method. The log-likelihood was −410.874, and AIC (Akaike's Information Criterion) was 833.748 which was useful in selecting predictors for regression and to find the order of the ARIMA model. Then, the BIC (Bayesian Information Criterion) was 851.931 which helped to get the normalization complete. It gives the efficiency of the trained model in terms of predicting the data. We have got a better normalization curve for the EEG data. RMSE (Root Mean Square Error) value was 2.834 for the signal range up to 100. mean squared error (MSE) value was 8.03. We have achieved a prediction accuracy of approximately 92%.

In order to justify that the ARIMA model was efficient in handling the input EEG data, we performed the computational modelling using LSTM and ANN algorithms for comparative analysis.  Figure 13 shows a comparison plot of the prediction errors among the models. We have used 3 primary metrics such as root mean squared error (RSME), mean absolute error (MAE), and mean squared error (MSE) to evaluate between the models. From the graph, we observed that the ARIMA model has reduced the RSME value by 60% compared to LSTM and 49% reduction was observed with respect to ANN. In terms of MAE value, the ARIMA has decreased the error by 80% with ANN and 30% with LSTM. Using the values of MSE, our model has performed well in reducing the error in the prediction against LSTM and ANN by 84% and 73%, respectively. Finally, we were able to conclude that the ARIMA model outperformed the ANN and LSTM models in terms of giving the least error prediction.

Therefore, when the EEG patterns of the normal sleep were changing, the ARIMA model displayed the changes on the signal patterns more efficiently. The abnormalities in the signal patterns would be analyzed by the healthcare specialist, and they can detect the likelihood for coma and the essential message would be triggered to the human. However, we faced a constraint while acquiring ECG data for this paper as there was no open-source ECG coma dataset available for training the prediction model, which we will attempt to focus in the future research work.

## 7. Conclusions

In this paper, we proposed an architecture to explore the EEG and ECG pattern for the sleep, awake, and comatose stage of a person. This helps the healthcare specialists to remotely monitor and mitigate the risks related to the human's health. The proposed architecture utilizes the benefits of HiLCPS and employs ARIMA to explore patterns that exist in the dataset. We used EEG dataset from an open-source community to conduct the experiment. To measure the efficiency of the ARIMA model, we performed comparative analysis with other deep learning algorithms such as LSTM and ANN. To the best of our knowledge, the proposed work achieved a greater prediction accuracy of the disease with less computational power compared to other deep learning algorithms.

## Figures and Tables

**Figure 1:** Inducing factors and consequences of coma.

**Figure 2:** Comparison of EEG patterns with each background activity [28].

**Figure 3:** EEG patterns during awake, 4 sleep stages, and anesthesia [29].

**Figure 4:** HRV against *R*-*R* intervals (millisecond) plotted over time (minutes) during the awake state, light NREM (stages 1 and 2), deep NREM (stages 3), and REM sleep [36].

**Figure 5:** Comparison of EEG patterns in (a) beta coma, (b) alpha coma, (c) theta coma, and (d) high-voltage delta coma [37].

**Figure 6:** ECG pattern on coma [38].

**Figure 7:** Human-in-the loop cyber-physical system correlation to the proposed architecture.

**Figure 8:** Proposed human-in-the-loop cyber-physical system in healthcare.

**Figure 9:** Sleep EEG signal.

**Figure 10:** Coma EEG signal.

**Figure 11:** ARIMA model result.

**Figure 12:** Prediction result.

**Figure 13:** Prediction error comparison among different models.

**Table 1:** Experimental setup.

Component	Specifications
Processor	Intel i5 9600k
Hard disk	Seagate 1 TB
GPU	RTX 2080
SSD	860 EVO 1 TB
Memory	32 GB DDR4 2666 MHz
Operation system	Windows 10 Professional
Computational software	Python 3.7
Interface	Pycharm

## Data Availability

The numeric data used to support the findings of this study are included in the article.

## Abbreviations

HiLCPS: Human-in-the-loop cyber-physical system
EEG: Electroencephalogram
ECG: Electrocardiogram
CPS: Cyber-physical system
IoT: Internet of Things
WSN: Wireless sensor network
CNN: Convolutional neural network
RSE: Refractory status epilepticus
PLEDS: Periodic lateralized epileptiform discharges
BIIPLEDS: Bilateral independent lateralized epileptiform discharges
GPEDS: Generalized periodic epileptiform discharges
BCI: Brain-computer interface
REM: Rapid eye movement
NREM: Nonrapid eye movement.
